The article "Facial Nerve Monitoring under Different Levels of Neuromuscular Blockade with Cisatracurium Besilate in Parotid Tumour Surgery" was retracted in 2024. Reasons: signs of a paper mill; suspected computer-generated content; unreliable results or conclusions; concerns about the data.

# Facial Nerve Monitoring under Different Levels of Neuromuscular Blockade with Cisatracurium Besilate in Parotid Tumour Surgery

**DOI:** 10.1155/2021/5655061

**Published:** 2021-07-13

**Authors:** Huimin Huang, Hong Jiang, Jinxing Liu, Jie Chen, Lin Qiu, Jiayi Wang, Wenhui Liu, Huan Chen

**Affiliations:** Department of Anesthesiology, Shanghai 9th People's Hospital, Shanghai Jiao Tong University School of Medicine, Shanghai, China

## Abstract

**Background:**

Anaesthesia can alter neuronal excitability and vascular reactivity and ultimately lead to neurovascular coupling. Precise control of the skeletal muscle relaxant doses is the key in reducing anaesthetic damage.

**Methods:**

A total of 102 patients with the normal functioning preoperative facial nerve who required parotid tumour resection were included in this study. Facial nerve monitoring was conducted intraoperatively. The surgeon stimulated the facial nerve at different myorelaxation intervals at TOF% (T4/T1) and T1% (T1/T0) and recorded the responses and the amplitude of electromyogram (EMG). Body movements (BM) or patient-ventilator asynchrony (PVA) was recorded intraoperatively.

**Results:**

In parotid tumour resection, T1% should be maintained at a range of 30 to 60% while TOF% should be maintained at a range of 20 to 30%. Analysis of the decision tree model for facial nerve monitoring suggests a partial muscle relaxation level of 30% < T1% ≤ 50% and TOF ≤ 60%. A nomogram prediction model, while incorporating factors such as sex, age, BMI, TOF%, and T1%, was constructed to predict the risk of BM/PVA during surgery, showing good predictive performance.

**Conclusions:**

This study revealed an adequate level of neuromuscular blockade in intraoperative parotid tumour resection while conducting facial nerve monitoring. A visual nomogram prediction model was constructed to guide anaesthetists in improving the anaesthetic plan.

## 1. Introduction

Anaesthesia can alter neuronal excitability and vascular reactivity and ultimately lead to neurovascular coupling [1]. Skeletal muscle relaxants are widely used in anaesthesia. However, numerous studies have linked skeletal muscle relaxants to neurovascular side effects [2, 3]. Therefore, precise control of the skeletal muscle relaxants dose is the key in reducing anaesthetic damage [4].

Facial nerve injury is a relatively common and major complication of parotidectomy that is disheartening to surgeons and the patients. Intraoperative facial nerve monitoring can significantly reduce postoperative facial nerve injury [5–8]. It is traditionally held that skeletal muscle relaxants should be avoided in general anaesthetic procedures requiring neuromonitoring. However, general anaesthesia without the use of skeletal muscle relaxants may aggravate anaesthetic damage and lead to intraoperative BM and PVA, affecting the surgical process [9]. To avoid BM/PVA, anaesthetists often need to increase the dose of intraoperative analgesics and sedative drugs. However, this may increase the risk of anaesthesia-related complications such as neurovascular injury, intraoperative circulatory depression, and delayed postoperative awakening.

In this study, nondepolarizing skeletal muscle relaxant, Cisatracurium besilate, was used in total intravenous anaesthesia during parotid tumour resection requiring facial nerve monitoring. The study is aimed at determining the appropriate level of muscular relaxation and providing a reference for general anaesthetic procedures requiring facial nerve monitoring by exploring the feasibility of facial nerve monitoring under partial muscular relaxation.

## 2. Materials and Methods

### 2.1. Basic Characteristics

This was a prospective study done between 2019 and 2020 at the Ninth People's Hospital. The study was approved by the Ethics Committee of the Clinical Trial Center of the Ninth People's Hospital of Shanghai Jiao Tong University (Ethics No. 2017-405-T302). Patients requiring parotid tumour resection who were classified under American Society of Anesthesiologists (ASA) grade I to II (*n* = 102) were selected for the inclusion to the study. Exclusion criteria are comprised of patients with Cisatracurium besilate allergy, facial palsy, or other neuromuscular diseases, history of diabetes mellitus, epilepsy, and craniotomy that may affect neuromonitoring. Anaesthesia was intravenously administered, with routine ECG monitoring, bispectral index (BIS) monitoring for the depth of anaesthesia, facial nerve EMG, and muscle relaxation monitoring (TOF%, T1%) carried out. Cisatracurium besilate was used intermittently during the operation. The surgeon recorded the facial nerve EMG at different levels of myorelaxation while stimulating the facial nerve or adjacent tissues to the operative area during the excision of the parotid tumour. BM and PVA were also recorded intraoperatively.

### 2.2. General Anaesthesia and Muscle Relaxation Monitoring

Patients admitted to the operating room underwent routine cardiac monitoring and received preoperative medication 30 min before the surgery. Before induction of the general anaesthesia, the Veryark-TOF muscle relaxation monitor (Willie's Ark, China) was connected to the ulnar nerve on the left upper forearm. The muscle tone sensor was placed at the tiger's mouth of the hand while the temperature sensor was placed at the inner thumb muscle and secured with an adhesive tape. The muscle relaxation monitoring was set up in the train-of-four stimulation (TOF) mode with one-minute repetitive stimulation time, and the TOF% (T4/T1) and T1% (T1/T0) values were recorded. In the induction of general anaesthesia, patients were sedated by intravenous administration of midazolam 0.05 mg/kg, fentanyl 2 *μ*g/kg, and propofol 2 mg/kg. T0 value and the appropriate stimulation current were determined. Cisatracurium besilate 0.15 mg/kg (3 × ED95) was then administered intravenously, and the tracheal tube was inserted. The BIS electrodes were connected to monitor the depth of anaesthesia. For the maintenance of general anaesthesia, continuous propofol 2-10 mg/(kg·h) and remifentanil 0.1-2 *μ*g/(kg·min) were administered with real-time regulation to maintain intraoperative vital signs, BIS between 40 and 60, and End-Tidal Carbon Dioxide (ETCO_2_) between 35 and 45. Single additional doses of Cisatracurium besilate 0.025 mg/kg (0.5 × ED95) were also given intraoperatively to maintain partial muscle relaxation in the following cases: (a) patients developed BM/PVA, (b) intraoperative electrokinetic stimulation of the patient's muscle twitching was too pronounced to interfere with the procedure, and (c) patients' TOF% or T1% was >91%.

### 2.3. Facial Nerve Monitoring

A Medtronic NIM-Neuro 3.0 neuromonitor (Medtronic Xomed, Inc., USA) was used to record the facial nerve EMG upon induction of general anaesthesia. Stimulating electrodes were inserted into the frontalis, orbicularis oculi, orbicularis orientalis, and chin muscles, while the grounding electrodes were inserted to the thorax and then connected to the mainframe of the facial nerve monitor. The facial nerve or adjacent tissues were stimulated with bipolar electrodes. To ensure accuracy of the facial nerve stimulation, the main trunk of the facial nerve or main branches, the mandibular margin branch and the temporal branch, was selected. Stimulation intensity was 0.20 mA, and the event threshold was 100 *μ*V. Facial nerve stimulation was considered positive at an EMG wave amplitude > 100 *μ*V and an abrupt rise in EMG changes.

### 2.4. Observation Parameters

Patients' facial nerve EMG responses and specific wave amplitude values were recorded at different muscle relaxation intervals. The TOF% (T4/T1) and T1% (T1/T0) were divided into eleven different muscle relaxation intervals, such as 0%, 1-10%, 11-20%, 21-30%, 31-40%, 41-50%, 51-60%, 61-70%, 71-80%, 81-90%, and 91-100%. Patients were continuously monitored for muscle relaxation. The facial nerve was stimulated intraoperatively at different intervals of TOF% and T1%, and the response to facial nerve monitoring was recorded and the wave amplitude of the EMG was recorded when there was a positive reaction. Patients were continuously observed for limb and swallowing movements, under different levels of muscle relaxation. The BM score was calculated by dividing stimulus with BM by stimulus without BM. The presence of autonomic respiratory waveform on the monitor and anaesthetic machine was recorded under different levels of muscle relaxation.

### 2.5. Statistical Analysis

Statistical analyses were done using R software (version 3.6.0). Visualization of the decision tree was done with the treeheater package, as described in a previous study [10]. The receiver operating characteristic curve (ROC) was used to assess the predictive accuracy of T1% and TOF% [11]. Nomogram was used to construct predictive models to assess the risk of BM/PVA. The calibration curve and C-index were further used to assess the predictive power of the nomogram [12, 13]. One-way ANOVA or two-tailed *t*-test was used to determine significance between groups. Values of *P* < 0.05 were considered statistically significant.

## 3. Results

### 3.1. Demographic and Clinical Characteristics

A total of 102 patients (48 males and 54 females) undergoing parotid mass resection were included in this study. All patients included in the study were in ASA classification grade I to II. Patients had a mean age of 44.49 ± 13.02 years, weight of 65.54 ± 13.51 kg, and height of 167.21 ± 8.62 cm.

### 3.2. T1% Relationship to the Optimal Dose of the Neuromuscular Relaxant

A histogram of BM/PVA and T1% is shown in Figures 1(a) and 1(b). The chi-square test revealed a significant correlation between T1% and BM/PVA (*P* < 0.001) (Figure 1(c)). Patients experienced significantly elevated BM/PVA at T1% ≥ 60%. The correlation between different intraoperative muscle relaxation conditions (T1%) and positive EMG reaction of the facial nerve was shown to be significant using chi-square analysis (*P* < 0.001) (Figures 1(d) and 1(e)). As shown in Figure 1(d), EMG monitoring of the facial nerve was largely unaffected at T1% > 30% when the muscle relaxation was maintained with Cisatracurium besilate in TIVA. This suggests that T1% should be controlled at a range of between 30 and 60% in parotidectomy.

### 3.3. TOF% Relationship to Neuromuscular Blockade Levels in Facial Nerve Monitoring

A histogram of BM/PVA and TOF% is shown in Figures 2(a) and 2(b). The relationship between different intraoperative muscle relaxation levels (TOF%) and the occurrence of BM/PVA was calculated using the chi-square test, which revealed a significant correlation (*P* < 0.001) (Figure 2(c)). Patients were shown to experience significantly elevated BM/PVA when TOF% ≥ 30%. The correlation between different intraoperative muscle relaxation levels (TOF%) and positive EMG reaction of the facial nerve using chi-square analysis was shown to be significant (*P* < 0.001) (Figures 2(d) and 2(e)). As seen in Figure 2(d), EMG monitoring of the facial nerve was largely unaffected at TOF% > 20% when muscle relaxation was maintained with Cisatracurium besilate in TIVA. This suggests that TOF% should be controlled at a range of 20 to 30% in parotidectomy.

### 3.4. ROC Curves of TOF% and T1% for Predicting the Effect of Facial Nerve Anaesthesia on Muscle Relaxation

As shown in Figure 3(a), the ROC curve had an AUC of 0.896 for TOF% and 0.947 for T1%, both close to 1. It can be concluded that the different intervals of TOF% and T1% values are ideal for determining the presence of BM/PVA, with T1% being relatively better than TOF%.  Figure 3(b) shows a ROC curve plotted against the facial nerve EMG showing an AUC of 0.909 for TOF% and 0.897 for T1%, which were also close to 1. It can be concluded that the different intervals of TOF% and T1% values are ideal for determining effectiveness of facial nerve monitoring. It is worth noting that the magnitude of facial nerve EMG values did not correlate linearly with TOF% and T1%. EMG amplitude values in most patients were below 1000 *μ*V and did not increase as the muscle relaxation lessened (Figure 3(c)).

### 3.5. Visualization of the Decision Tree

Decision trees were drawn to guide visualization for better clinical application. As shown in Figure 4(a), the decision tree-heat map for predicting BM/PVA occurrence during surgery reflects that T1% ≤ 50% does not result in BM/PVA, while TOF% > 60% is a high-risk factor for BM/PVA occurrence. Therefore, in parotidectomy, T1% should be maintained ≤50% and TOF ≤ 60%. As shown in Figure 4(b), a decision tree-heat map for predicting the incidence of a positive EMG response of the facial nerve during surgery revealed a good positive EMG reaction of the facial nerve at T1% > 30%. Women were seen to be less likely to have a negative EMG reaction of the facial nerve compared to men. In conclusion, 30% < T1% ≤ 50% and TOF ≤ 60% should be maintained.

### 3.6. A Visual Nomogram Prediction Model

In clinical practice, the final anaesthetic outcome may be influenced by several factors. Therefore, a visual nomogram prediction model was constructed to predict the likelihood of patients developing BM/PVA during surgery, while incorporating factors such as sex, age, BMI, TOF%, and T1% (Figure 5(a)). The specific parameters of the visual nomogram prediction model are shown in Table 1. The overall prediction performance of the prediction model was good as the solid line was very close to the dashed line in the calibration curve (Figure 5(b)). The C-index was 0.959 (95% CI, 0.935-0.982, entire cohort) (Table 2). The model also had a good internal validation. This model shows that a low BMI, young age, and female gender were more likely to be associated with BM/PVA during surgery, and patients should be anaesthetized at an increased depth.

## 4. Discussion

In this study, we explored the optimal cut-off value for neurovascular anaesthesia on muscle relaxation in local surgery involving parotid tumour resection. Appropriate level of muscle relaxation should be maintained in parotidectomy with facial nerve monitoring. TOF% and T1% are useful markers of the degree of muscle relaxation during facial nerve monitoring. We recommend a partial muscle relaxation level of 30% < T1% ≤ 50% and TOF ≤ 60% for facial nerve monitoring, and the operator should be aware of the presence of a negative EMG reaction of the facial nerve when dealing with female patients. Construction of a visual nomogram prediction model was done to guide anaesthetists in the anaesthetic plan.

Due to the proximity of the anatomical structures to the facial nerve, the use of facial nerve monitoring can significantly reduce the incidence of postoperative facial nerve injury in a large number of craniomaxillofacial surgical operations including auditory neuroma at the base of the skull, middle ear, and parotid area surgery [5–8, 14, 15]. Facial nerve monitoring tools have resulted in increased use of facial nerve monitoring thus avoiding or reducing the chances of facial paralysis in patients undergoing surgery. The use of skeletal muscle relaxants in general anaesthesia may affect EMG or contraction of the facial muscles by reducing the transmission of electrical signals from the neuromuscular junction thus affecting facial nerve monitoring. For this reason, surgeons recommend that skeletal muscle relaxants be avoided during general anaesthetic procedures requiring facial nerve monitoring. However, avoiding use of skeletal muscle relaxants in general anaesthesia requires anesthesiologists to increase the dose of intraoperative analgesics and sedative drugs so as to avoid BM and PVA. This increases the risk of intraoperative circulatory depression, delayed postoperative awakening, hypothermia, and other anaesthetic complications. The use of a higher dose of the analgesic, remifentanil, under general anaesthesia was shown to decrease the incidence of intraoperative BM from 44 to 20%. However, the highest dose of remifentanil (0.21 mg/kg·min) did not completely prevent BM and was associated with increased intraoperative hypotension and bradycardia and circulatory depression [16]. Maintaining partial muscle relaxation in general anaesthesia has been shown to be a more effective strategy. In recent years, skeletal muscle relaxants have been used during general anaesthesia in a variety of procedures requiring neuromonitoring to induce a partially muscle relaxed state [17–21].

In this study, the nondepolarizing skeletal muscular relaxant, Cisatracurium besilate, was used. The study revealed that facial nerve monitoring could be effectively performed under partial muscle relaxation. The suitable range of partial muscle relaxation was determined as TOF% between 20 and 30% or T1% between 30 and 50%. Noteworthily, the TOF% value is considered a classical indicator of the degree of muscle relaxation. In this study, a positive EMG reaction in facial nerve monitoring was seen in some patients in muscle relaxation recovery with a TOF% of 0 and a partial recovery at T1%. There was no reaction to facial nerve stimulation in all patients when T1% was 0. T1% was more sensitive in facial nerve monitoring during the initial phase of myosin recovery which is consistent with the findings of Chung et al. Chung et al. recommended using T1% as the control target in determining the required degree of partial muscle relaxation when monitoring facial muscle lateral spread response (LSR) during microvascular decompression as opposed to using TOF% [21]. Additionally, surgeons are often interested in the amplitude of the facial nerve EMG when isolating the facial nerve. The present study shows that the amplitude of the facial nerve EMG does not increase linearly as the muscle relaxation is restored. The EMG response values may be more relevant to individual differences than the degree of muscle relaxation recovery.

There are several other factors that affect facial nerve monitoring. Firstly, the use of inhalation drugs in general anaesthesia may inhibit neuromuscular function and have synergistic effects with skeletal muscle relaxants, thus affecting recovery [22, 23]. To control this, general anaesthesia was maintained under TIVA. The correlation between maintenance and recovery time from muscle relaxation and facial nerve monitoring needs to be confirmed by further clinical studies. Secondly, there has been opposition to carry out facial nerve monitoring during parotid surgery, due to false-positive and false-negative results occasioned by unfamiliarity with facial nerve anatomy, mechanical failure, and anaesthetic drugs [5, 24–26]. When using a facial nerve monitor during parotidectomy and stimulating the facial nerve with a bipolar electroacupuncture needle, if the anatomy of the stimulated facial nerve branch is abnormal, the muscle into which the electrode is inserted is not within the innervation of the stimulated nerve, resulting in a false-negative result. In this study, the surgeon chose to stimulate mainly the main trunk of the facial nerve or its main branches, the mandibular marginal branch and the temporal branch, to avoid false negatives. Patients with superficial location of the tumour with the inaccessible target nerve or with excessive intraoperative bleeding were excluded from the study.

This study had some limitations. (1) Due to the limited number of parotid tumour cases, the line graphs could not be externally validated, and thus, another study with a large sample size is required. (2) The study population was all Asian, and thus, the study findings may not be generalizable to other populations. (3) Construction of the predictive models needs to be enriched further. In future studies, we need to collect more data and further refine the multicentre study to construct more accurate predictive models.

## 5. Conclusion

In summary, we explored the optimal cut-off value for the effect of neurovascular anaesthesia on muscle relaxation in local parotid tumour surgery with facial nerve monitoring. TOF% and T1% are good indicators of the degree of muscle relaxation during facial nerve monitoring, with T1% being more sensitive compared to TOF%. We recommend a partial muscle relaxation level of 30% < T1% ≤ 50% and TOF ≤ 60% for facial nerve monitoring, and the operator should be aware of the presence of a negative EMG reaction of the facial nerve when dealing with female patients. A visual nomogram prediction model is also available to provide the anaesthetist with a detailed guide to improve the anaesthetic plan.

## Figures and Tables

**Figure 1:** Relationship between T1% and the degree of muscle relaxation with skeletal muscle relaxants in facial nerve monitoring: (a) T1% and body movement score relationship; (b) T1% and patient-ventilator asynchrony relationship; (c) estimated T1% with/without BM/PVA; (d) T1% and positive facial nerve EMG reaction relationship; (e) comparison of estimated T1% between positive EMG reaction and negative EMG reaction.

**Figure 2:** Relationship between TOF% and the cut-off value for the effect of facial nerve anaesthesia for muscle relaxation: (a) the relationship between TOF% and body movement score; (b) the relationship between TOF% and patient-ventilator asynchrony; (c) comparison of estimated TOF% with/without BM/PVA; (d) the relationship between TOF% and positive EMG reaction of the facial nerve; (e) comparison of estimated TOF% between positive EMG reaction and negative EMG reaction.

**Figure 3:** ROC curves of TOF% and T1% for predicting the effect of facial nerve anaesthesia on muscle relaxation: (a) ROC curve of TOF% and T1% for body movement or patient-ventilator asynchrony; (b) ROC curve of TOF% and T1% for body movement or positive EMG reaction of the facial nerve; (c) correlation of EMG values with TOF% and T1%.

**Figure 4:** Visualization of the decision tree. (a) A decision tree-heat map for predicting the occurrence of BM or PVA during surgery. MRVC: movement or ventilation confrontation has occurred; ASA: American Society of Anesthesiologists. (b) A decision tree-heat map for predicting a positive EMG response of the facial nerve during surgery. EMG: electromyogram. Note: the heat map colours present the relative value of a sample compared to the rest of the group.

**Figure 5:** A visual nomogram prediction model. (a) Nomogram prediction model for predicting the occurrence of BM or PVA during surgery. (b) Calibration curve of the BM/PVA model for predicting the occurrence of BM/PVA during surgery. The closer the solid line to the dashed line, the better the predictive power.

**Table 1:** Chart showing the prediction factors.

Variable	Prediction model		
	*β*	Odds ratio (95% CI)	*P* value
Intercept	0.034	0.001 (0-0.119)	0.007
TOF%	-0.059	1.396 (1.123-1.768)	0.004
T1%	-0.678	2.633 (1.909-3.888)	*P* < 0.001
Sex (male)	2.189	0.657 (0.203-2.053)	0.472
Age (years)	-2.003	0.983 (0.944-1.022)	0.391
BMI	-0.001	0.88 (0.723-1.048)	0.172

Note: *β* is the regression coefficient.

**Table 2:** C-index of the nomogram prediction model.

Features	C-index (95% confidence interval)
Entire cohort	0.959 (0.935-0.982)
Train set	0.977 (0.957-0.997)
Validation set	0.905 (0.84-0.97)

## Data Availability

Raw data are available on request from the corresponding author.

## Abbreviations

AUC: Area under the curve
ASA: American Society of Anesthesiologists
BM: Body movement
BIS: Bispectral index
EMG: Electromyogram
PVA: Patient-ventilator asynchrony
ROC: The receiver operating characteristic curve
TOF: Train-of-four stimulation
TIVA: Total intravenous anaesthesia.
